# Advances in Experimental and Clinical Research of the Gouty Arthritis Treatment with Traditional Chinese Medicine

**DOI:** 10.1155/2021/8698232

**Published:** 2021-10-20

**Authors:** Huan Liang, Pin Deng, Yu-Feng Ma, Yan Wu, Zhan-Hua Ma, Wei Zhang, Jun-De Wu, Yin-Ze Qi, Xu-Yue Pan, Fa-Sen Huang, Si-Yuan Lv, Jing-Lu Han, Wen-Da Dai, Zhaojun Chen

**Affiliations:** ^1^School of Graduates, Beijing University of Chinese Medicine, Beijing 100029, China; ^2^Department of Hand and Foot Surgery, Beijing University of Chinese Medicine Third Affiliated Hospital, Beijing 100029, China

## Abstract

Gouty arthritis (GA) is a multifactorial disease whose pathogenesis is utterly complex, and the current clinical treatment methods cannot wholly prevent GA development. Western medicine is the primary treatment strategy for gouty arthritis, but it owns an unfavorable prognosis. Therefore, the prevention and treatment of GA are essential. In China, traditional Chinese medicine (TCM) has been adopted for GA prevention and treatment for thousands of years. Gout patients are usually treated with TCM according to their different conditions, and long-term results can be achieved by improving their physical condition. And TCM has been proved to be an effective method to treat gout in modern China. Nevertheless, the pharmacological mechanism of TCM for gout is still unclear, which limits its spread. The theory of prevention and treatment of gout with TCM is more well acknowledged in China than in abroad. In this article, Chinese herbs and ancient formula for gout were summarized first. A total of more than 570 studies published from 2004 to June 2021 in PubMed, Medline, CNKI, VIP, Web of Science databases and Chinese Pharmacopoeia and traditional Chinese books were searched; the current status of TCM in the treatment of GA was summarized from the following aspects: articular chondrocyte apoptosis inhibition, antioxidative stress response, inflammatory cytokine levels regulation, uric acid excretion promotion, immune function regulation, uric acid reduction, and intestinal flora improvement in subjects with gout. The literature review concluded that TCM has a specific curative effect on the prevention and treatment of GA, particularly when combined with modern medical approaches. However, lacking a uniform definition of GA syndrome differentiation and the support of evidence-based medicine in clinical practice have provoked considerable concern in previous studies, which needs to be addressed in future research.

## 1. Introduction

Gout is a crystal-related disease aroused by the sedimentation of monosodium urate (MSU), directly related to hyperuricemia caused by decreased uric acid excretion or purine metabolic disorders [1]. Gout incidence rate and prevalence have risen steadily over the past few decades due to lifestyle changes, westernized diets, and an aging population [2]. Typical acute gouty arthritis is more common in middle-aged, older men, and obese postmenopausal women. It is usually manifested as redness, bright, and significant tenderness in the single affected joints, especially when the first metatarsophalangeal joint is involved [3]. A considerable part of the global population experiences gout every year [4]. According to World Health Organization (WHO) estimates, 3.9% of the people in the world suffer from gout [5]. Gout owns multiple risk factors such as obesity, coronary heart disease, hypertension, diabetes or glucose intolerance, and lipid metabolism disorders. Acute episodes of arthritis, chronic joint injury, and joint malformations can decrease the living quality and cause disablement in some severe cases [6, 7].

Western medicine is the primary treatment strategy for gout (such as uric acid-lowering drugs, pain relief, primary disease treatment, physical therapy, and surgical treatment). These drugs have certain adverse effects on liver, kidney, and gastrointestinal tract, thus influence patients' treatment compliance [8]. However, the overall prognosis of gout is still not optimistic. TCM is considered a treasure trove of clinical practice for thousands of years and a significant contributor to global medical care. TCM originated in ancient China. Therefore, it has been applied to the prevention and treatment of gout for many centuries in China. Chinese medicine, with unique efficacy, has the long clinical practice and a lot of clinical experience in preventing and treating gout [9], No matter TCM is used alone or combined with other therapies, it is the most commonly used complementary and alternative medicine (CAM) in modern China and is beneficial to subjects with gout [10]. TCM contains rich culture and literature, which is mainly reflected in two parts: Chinese medicine itself and the theoretical system of TCM. “Disease prevention” is the principle of TCM for disease treatment. TCM has emphasized the prevention and treatment of diseases. For the prevention and treatment of gout disease, we can combine the theory of “treating pre-disease” and “the principle of a holistic view of TCM” according to the characteristics of the development of the disease.

As early as 2000 years ago, the authoritative work of TCM “Huangdi Neijing·Suwen” made a detailed discussion on the etiology, pathogenesis, syndrome classification, and prognosis of gout [11]. Etiology is the core of TCM theory, which studies gout syndrome based on holism. According to the theory of TCM, gout is associated with congenital deficiency and dysfunction of the spleen and kidney. Holism holds that the spleen is the root of after birth and the source of qi and blood, which transports the essence of water and grain to nourish the whole body. The kidney is often considered as the congenital foundation, which can store substances and regulate water metabolism [12]. TCM practitioners in China emphasize the intrinsic balance of the body. Consequently, TCM works not just by treating gouty arthritis itself but also by curing the patient as a whole in an indirect way [13].

For GA, it is proven that many effective fang-ji (formulations) can clinically delay gout's progress and prevent the occurrence of it. The fang-ji was designed according to the theory of spleen and kidney disorders and qi and blood in TCM [14]. In this review, the Chinese herbs and ancient formulas with remedial effects on GA were summed up first. Then, the current research situations of TCM in modern medicine were analyzed, coming up with existing issues in the development of TCM. Lastly, the future of TCM in the circumstance of integrated medicine and precision medicine was concluded. After the review was completed, it was convinced that TCM is a progressive GA therapy despite its development since ancient times; it has curative effects, although the controversy still exists. The theory of TCM also needs to be precisely analyzed and confirmed by systematic research methods.

## 2. History of TCM for GA Prevention and Treatment

Classical TCM formulas applied to prevent and treat gouty arthritis for thousands of years are the most popular utilization of TCM. Gout originated in the late Western Han Dynasty. In the ancient books about TCM, there is no clear concept of “gouty arthritis” as it is in the modern medicine. The symptoms and pathogenesis of “Li-Jie disease,” “white tiger disease,” and “gout” in TCM have many similarities with gouty arthritis. Gouty arthritis belongs to the category of “Bi syndrome” in TCM, and the TCM disease name “Bi syndrome” was observed for the first time in Huangdi's Internal Canon (Huang Di Nei Jing in Chinese) [15]. In TCM ancient literature, the scope of “Bi syndrome” is extensive, which includes many Western medicine diseases.

Following Huangdi's Internal Canon, Zhang Zhongjing of the Han Dynasty was the first to elaborate gout systematically. Zhang Zhongjing discussed gout treatment in “jin-gui-yao-lue” and proposed using “Ramulus Cinnamomi, Paeoniae and Anemarrhenae decoction” to treat gout syndrome of wind-damp associated with pathogenic heat. “Wu-tou decoction” treats gout syndrome of cold dampness. Since the Han Dynasty (over 2000 years ago), TCM physicians inherited and developed Zhongjing's doctrine and gained a deeper and more comprehensive understanding of the causes and mechanisms of Li-Jie disease, and the therapeutic methods and typical recipes were more abundant [16].

Cao Yuanfang of the Sui Dynasty emphasized the effects of deficient qi and blood and alcohol consumption on gout in his “General Treatise on the Cause and Symptoms of Diseases,” stressing the deficiency in origin and excess in the superficiality of Bi's disease [17]. Wang Tao of the Tang Dynasty emphasized that the pathogenesis of gout was “dampness and heat, phlegm hinder the meridians” in his “Wai-tai-mi-yao,” which is basically consistent with the view of the Huangdi's Internal Canon (Huang Di Nei Jing in Chinese) [18]. Zhu Danxi, one of the four schools of the Jin-yuan Dynasty, officially proposed the name of gout. In his book “Danxi's Mastery of Medicine·Gout,” he pointed out that the pathogenesis of gout is “phlegm, wind-heat, wind-damp, blood-insufficiency, blood heat, and blood stasis, which are blocked in the meridians and collaterals [19].

The primary treatment is related to the specific pathogenesis of the patient. For people with blood-insufficiency symptoms, Chuanxiong Rhizoma (Chuan xiong) and *Angelicae Sinensis Radix* (Dang gui) are mostly used accompanied by Persicae Semen (Tao ren), Carthami Flos (Hong hua), and Radix Clematidis (Wei ling xian). In case of people with damp evil retention syndrome, consider adding *Atractylodes Lancea* (Cang zhu), *Atractylodes Macrocephala Koidz* (Bai zhu), and Bamboo Juice (Zhu li) based on Erchen decoction to invigorating the spleen and removing dampness. In the case of phlegm blockage, it is considered to add *Scutellariae Radix* (Huang qin), Notopterygii Rhizoma Et Radix (Qiang huo), and *Atractylodes Lancea* (Cang zhu) to Er Chen decoction to dissolve phlegm and clear the collaterals.

For patients with blood stasis symptoms, *Saposhnikoviae Radix* (Fang feng) and Notopterygii Rhizoma Et Radix (Qiang huo) are added to Siwu decoction to activate blood circulation and dissipate blood stasis. For patients with obvious blood stasis symptoms, add *Scutellariae Radix* (Huang qin) and *Phellodendri Chinrnsis Cortex* (Huang bai) to Si Wu Tang to nourish the blood, promote blood circulation, clear heat, and dry dampness. During the Ming and Qing dynasties, Wang Kentang's classic work “zheng-zhi-zhun-sheng” attributed the cause of gout to wind-dampness invading the kidney meridian, causing stagnation in the blood vessels [20]. Zhang Jingyue pointed out in his “Jing-Yue-Quan-Shu” that the wandering arthritis syndrome in TCM is gout [21]. Wang Qingren of the Qing Dynasty proposed a Chinese medicine prescription to treat gout by invigorating Qi, promoting blood circulation, and creating a new way of thinking for clinical practice in his “Yilin Gaicuo” [22].

Zhu Liangchun, a modern physician, believes that the pathogenesis of gout is caused by the dysmetabolism of spleen and kidney metabolic disorders, which leads to turbid damp originating from interior blood stasis and obstruction of main and collateral channels [23]. In the acute attack phase, it is recommended to use Smilacis Glabrae Rhixoma (Tu fu ling) and Dioscoreae Septemlo Bae Rhizoma (Bixie) with a significant dose to clearing away heat, eliminating dampness, and discharging phlegm turbidity. For patients with apparent joint redness and swelling, it is recommended to use *Radix Rehmanniae* (Sheng Di), *Gypsum rubrum* (Han shui shi), *Anemarrhenae Rhizoma* (Zhi mu), and *Cape buffalo* (Shui niu jiao) to clear away heat and dredge collaterals.

For patients with obvious pain symptoms, add scorpion (Quan xie), centipede (Wu gong), and Corydalis Rhizoma (Yan hu suo) to disperse stasis and relieve pain. If the disease progresses in chronic or intermittent stage, *Raw Atractylodes Macrocephala Koidz* (Sheng bai zhu), *Poria cocos* (Fu ling), Fructus Ligustri Lucidi (Nv zhen zi), and *Polygoni Multiflori Radix* (He shou wu) can regulate the spleen and kidney. The ancient Chinese medical literature on preventing and treating gout is very plentiful and has provided valuable experience for later generations of physicians to study gouty arthritis (Figure 1). Based on the experience of our predecessors and modern medical methods, a more in-depth study of gouty arthritis can be conducted.

## 3. Therapeutic Effect Stimulated the Development of TCM for GA in Ancient China

### 3.1. Herbs for Prophylaxis and Treatment of GA

Herbal medicines include thousands of plants species. They are used for GA treatment, and many of them are widely used. Single Chinese medicine is mainly used to clear heat and promote dampness in treating gout. The following ten Chinese herbal medicines are the most commonly used ones *Coix Seed*(Yi ren), *Phellodendri Chinrnsis Cortex* (Huang bai), *Atractylodes Lancea* (Cangzhu), *Plantaginis Semen* (Che qian zi), *Alisma Orientale* (Ze xie), Chuanxiong Rhizoma (Chuan xiong), Achyranthis Bidentatae Radix (Niuxi), Polygoni Cuspidati Rhizoma Et Radix (Hu zhang), *Saposhnikoviae Radix* (Fang feng), and Radix Angelicae Biseratae (Du huo) influence jian-pi-li-shi, huo-xue-hua-yu, and qing-re-jie-du; the detailed information is shown in Table 1.

### 3.2. Herbal Formulas for the Prophylaxis and Treatment of GA

Herbal formulas are the most popular application of TCM, and some typical herbal formulas have significantly prophylactic and therapeutic effects on GA. TCM can benefit patients through treatment based on syndrome differentiation, which is the characteristic and advantage of Chinese medicine. TCM treats gouty arthritis with great emphasis on the causative factors of “dampness” and “heat [24].” Si-miao-tang and Dang-gui-nian-tong-fang are herbal formulas used for restraining gouty arthritis through invigorating the spleen and dispelling dampness. Invigorating the spleen is an essential principle for GA treatment, and Simiao decoction is a notable herbal formula for invigorating the spleen to remove dampness and for detoxification.

Straightly removing pathogenic elements is another vital principle to treat GA with herb-ju-zhi-zi-cha-fang. *Smilacis Glabrae Rhixoma* (Tu fu ling) and *Dioscoreae Septemlo Bae Rhizoma* (Bixie) are the classical herbal composition to treat GA by removing dampness and detoxification in addition to conditioning therapy, such as Si-huang-san and Ju-zhi-dihuang-wan. After analyzing the literature obtained through searching, it was found that the treatment principle with TCM prescriptions for the treatment of gouty arthritis mainly was invigorating the spleen and removing dampness, clearing away heat, and detoxifying; the prescriptions that appeared frequently were summarized and classified according to the mentioned treatment principle. Due to content limitations, Table 2 only lists the most common and classic prescriptions for the treatment of gouty arthritis. The details are illustrated in Table 2.

### 3.3. The Disadvantages of TCM Theory and Chinese Medicine

The theory of TCM is not broadly accepted, which is the main obstacle to the modernization of TCM. Practices of TCM depend on the integration of TCM theory and individual experiences of physicians. The pharmacological mechanism of Chinese medicine for treating gout is still unclear, and it still needs to be thoroughly explored and studied whether Chinese medicine has effective methods to promote the dissolution and removal of urea salt deposits. Therefore, molecular and cellular biology in modern medicine have offered valuable perspectives for the mechanisms of GA and provided anti-inflammatory strategies. Although Chinese medicine has been documented and demonstrated to be available for the treatment of GA [25–27], the critics still indicate that the toxicity of Chinese medicine (CHM) is indistinct [28]. Consequently, exploring the molecular signal transduction mechanism of CHM and removing toxic components may help to increase the acceptance of TCM in modern society [29].

## 4. Research Status and Application of Chinese Medicine for GA in Current Medicine

### 4.1. GA Treatment with Chinese Medicine

The curative rate of GA is not satisfactory. In China, TCM has been used to prevent and treat gouty arthritis for a long time and is regarded as an available disease-preventing method [30]. TCM treatment of gout has the effect of lowering uric acid and can effectively inhibit inflammation, relieves gout symptoms, avoids recurrence, and avoid the potential risk of low serum uric acid (SUA) controlling. One of the clinical trials showed that TCM formula named Skin-patch of Xin Huang Pian, which mainly consisted of *Panax Notoginseng* (San Qi), *Concha Margaritifera Usta* (Zhen Zhu Ceng Fen), Herba Sarcandrae (Zhong Jie Feng), *Urena lobata Linn* (Xiao Fan Tian Hua), and *calculus bovis arti-factus* (Ren Gong Niu Huang) seemed to be efficacious and safe to alleviate joint symptoms of patients with acute gouty arthritis. The mechanism might be C-reactive protein and ESR decreasing [31]. RBXG formula stemmed from “Bixie Fenqing Yin” in “Medical Insights” have been demonstrated to reduce the risk of acute gouty arthritis recurrence. The classic decoction such as “Yellow-dragon Wonderful-seed Formula” and Simiao Pill is also efficacious for uric acid, erythrocyte sedimentation rate, and other inflammatory factors and have a clinical efficacy for gout patients [32, 33].

### 4.2. Anti-GA Therapy with Chinese Medicine

TCM is usually applied as an herbal formulation clinically based on TCM theory. Chinese medicine has unique advantages in preventing and treating gout due to its “multitarget” effect and has achieved good results in the treatment of gouty arthritis in recent years. Shi et al. reported 29 cases of gout patients with dampness heat turbid blood stasis syndrome who were treated with private (self-prescribed) herbal formula, and it showed that the levels of inflammatory factors such as Interleukin-1beta (IL)-1*β*, IL-6, Visual Analogue Scale (VAS) score, and Tumor necrosis factor (TNF)-ɑ were significantly decreased [34]. Wang et al. found that the incidence of the adverse reaction of Chuanhu antigout mixture was lower than that of colchicine treating acute gouty arthritis. In addition, Chuanhu antigout mixture also had the function of protecting kidney and renal function [35]. Combined treatment is more familiar in clinic practice for GA patients. Ren et al. found that the allergic risk for acute gouty arthritis patients treated with external application of compound Qingbi granules combined with oral loxoprofen sodium was lower than that treated with Diclofenac Diethylamine Emulsion externally [36], and the adverse reactions were reduced and the curative effects were improved after Qinbi granules combined with Indomethacin [37], colchicine or Celecoxib [38] and allopurinol tablet [39].

### 4.3. Patients' Symptoms Improve with Chinese Medicine

The followings are the most common Chinese medicines used for swollen joint and higher skin temperature treatment: *Phellodendri Chinrnsis Cortex* (Huang bai), *Coicis semen* (Yi ren), *Anemarrhenae Rhizoma* (Zhi mu), Talc (Hua shi); the most commonly used Chinese medicines for arthritis pain: Aconiti Lateralis Radix Praeparata (Wu tou), Curcumaelongae Rhizoma (Jiang huang); and the most widely used Chinese medicines for gouty tophi: Radix Clematidis (Wei ling xian), Cinnamomi Ramulus (Gui zhi), and Lycopi Herba (Ze lan) [40]. Gouty tophi is also a common complication of advanced gouty arthritis. External application of compound Qingbi granules can effectively relieve pain and reduce synovium thickness caused by arthritis. Meanwhile, external application of Chinese herbal compounds can also avoid adverse effects, reducing GA patients' reliance on analgesic medicine [41]. External application of compound TCM to the affected area or acupuncture point can directly work on the affected area, reducing swelling and relieving pain and improving the clinical symptoms and signs of patients with acute gouty arthritis (AGA) significantly [42]. The clinical trial results showed that Chinese medicine combined with cupping therapy had satisfactory results in treating 34 patients with gouty arthritis. It was very effective in improving Budzyuski pain index, lowering blood uric acid, and lowering joint swelling index [43]. The meta-analysis of the compound TCM Simiao San treating gouty arthritis showed that Simiao San, as a traditional Chinese medicine decoction, can improve the clinical symptoms and signs of patients with AGA [44].

## 5. Research Status of Anti-GA Mechanisms in TCM

### 5.1. Various Herbal Formulas Are Generally Illustrated in the Theory of TCM

Herbal medicine has many active ingredients. Many herbal formulations and their active ingredients have significant effects on articular chondrocytes apoptosis inhibition, anti-inflammation, antioxidation stress reaction, inflammatory cytokine levels regulation, uric acid excretion promotion, immune function regulation (cellular immunity regulation), uric acid levels reduction and intestinal flora improvement for gout patients [45–48], body resistance enhancement [49], purine metabolism regulation [50], renal damage prevention for gout patients, etc. [51] (Figure 2).

### 5.2. Articular Chondrocyte Apoptosis Inhibition

Gouty arthritis is characterized by joint inflammation and uncontrolled articular chondrocytes apoptosis. Articular chondrocytes apoptosis inhibition is a new method for the treatment of gouty arthritis. Formulas such as Jiawei Simiao powder [52] and Guizhi Shaoyao Zhimu decoction [53] and herbs including *Phellodendri Chinrnsis Cortex* (Huang bai) [54] and *Rhizoma Atrac-tylodis Lanceae* (Cang zhu) [55] can significantly inhibit articular chondrocytes apoptosis and have an antigout effect. The compounds isolated from *Radix Rhei Et Rhizome* (Da huang) [56] and *Stephaniae Tetrandrae Radix* (Fang ji) [57] can inhibit the inflammatory reaction of cells and regulate the immunity and metabolism of the human body. Simiao pill can inhibit articular chondrocytes apoptosis and improve cartilage lesions by reducing IL-1*β* expression, upregulating B-cell lymphoma (Bcl)-2 gene expression, and downregulating Bax gene expression [58]. Compound TCM with the function of clearing away heat, promoting diuresis, and dredging collateral methods may treat acute gouty arthritis by promoting apoptosis, inhibiting cell proliferation, and blocking cell cycle of fibroblast-like synoviocytes (FLS) to alleviate the inflammatory reaction regionally [59].

### 5.3. Antioxidation Stress Reaction

Oxidative stress refers to the state of imbalance between oxidative and antioxidative effects in the body, which tends to be oxidized, resulting in the inactivation of antioxidant (superoxide dismutase (SOD), glutathione peroxidase (GSH-Px), reduced glutathione, etc.) and aggravation of joint tissue damage [60]. Many kinds of Chinese medicine and effective ingredients have anti-inflammatory, antioxidant, and other pharmacological effects [61]. Tongfeng Kangning formula [62] and Zisheng Shenqi Pill can also relieve the oxidative stress state of the body and protect the joints from damage [63]. Quercetin [64] and papaya extract [65] can increase the activity of GSH-Px and superoxide dismutase (SOD) in GA animal model, reduce the level of malondialdehyde (MDA), and improve joint tissue damage through antioxidant effect. Resveratrol [66] is a polyphenol compound in Veratrum, which can regulate oxidative substances and reduce oxidative stress by activating Nrf2-mediated induction of heme oxygenase-1 (Nrf2/HO-1) signaling pathway. The ethanol extract of Chinese medicinal materials *Gentiana macrophylla* [67] can upregulate the expression of Sirtuin1 (SIRT1) and p53 protein acetylation (ac-p53) and downregulate the expression of p53 and MicroRNA 34a (miR-34a) protein in GA rats by regulating the SIRT1/p53 signaling pathway, so as to regulate antioxidants and reduce the oxidative damage to the body. Herba Ephedrae Sinicae (Mahuang) can remove reactive oxygen species (ROS) and has an obvious antioxidant effect [68].

### 5.4. Inflammatory Cytokine Levels Regulation

The inactivation of anti-inflammatory factors and the release of proinflammatory factors play an important role in the inflammatory response. Excessive release of inflammatory factors can induce a large number of neutrophils to infiltrate into the joint cavity and stimulate the activation of neutrophils, causing tissue inflammation [69]. The chemical components of TCM can regulate inflammatory cytokines. Berberine isolated from *Coptidis Rhizoma* (Huanglian) can inhibit the production of LPS (lipopolysaccharide)-mediated IL-1*β* and swelling of monosodium urate (MSU) mediated paw by blocking NOD-like receptor (NLR) family, pyrin domain-containing protein 3 (NLRP3) signaling pathway [70]. The ethanol extract of Rhizoma Dioscoreae Nipponicae (Chuanshanlong) can act on MAPK/JNK pathway and inhibit the secretion of inflammatory factors in GA rats [71]. Emodin can reduce the release of inflammatory factors by inhibiting the activation of extracellular signal regulated kinase (ERK) 1/2 and p38 mitogen-activated protein kinase (MAPK) signaling pathways [72]. Gallic acid can inhibit the migration of MSU-induced macrophages and neutrophils to synovitis by inhibiting the activation of NLRP3 inflammasomes and apoptosis of nuclear factor erythroid-2 related factor 2 (Nrf2) signals [73]. Chinese Medicine Huzhen Tongfeng Formula(HZTF) can downregulate cyclooxygenase (COX) 1, COX-2, and 5-lipoxygenase, inhibit gouty arthritis cell infiltration significantly, improve the swelling of the affected joints, and increase pain threshold by inhibiting the inflammatory mediators and the arachidonic acid metabolism [74]. Simiao decoction has the effect of reducing blood uric acid levels, reducing myeloperoxidase (MPO), xanthine oxidase (XOD), adenosine deaminase (ADA) activity, and alleviating gout-related symptoms (such as foot swelling and pain). In addition, it can also reduce certain specific proinflammatory cytokines in serum, including IL-1*β*, IL-9, interferon (IFN) g, macrophage inflammatory protein (MIP) 1a, and MIP-1b [75].

### 5.5. Uric Acid Excretion Promotion

It has been reported that *Achyranthis Bidentatae Radix* (Niuxi) can promote the excretion of uric acid, improve cellular and humoral immunity, as well as nonspecific immune function [76]. Fucoidan can promote uric acid excretion and relieve symptoms of uric acid nephropathy (UAN) by upregulating the expression of protein kinase A (PKA) and organic cation transporter 2 (OCT 2) in the kidney tissue surface [77]. Verbascoside is a phenylethanoid glycoside in *Plantago asiatica*, and it has been proved that it can inhibit XOD activity and decrease the expression of uric acid transporter 1 (URAT1) and glucose transporter (GLUT) 9 protein, reducing the production of uric acid and promoting the excretion of uric acid [78]. Eucommiae cortex alcohol extract [79] and anthocyanin [80] can enhance the expression of ATP-binding cassette subfamily G member 2 (ABCG2), OAT1, and organic anion transporter (OAT3) protein in hyperuricemia (HUA) and GA animal models and accelerate uric acid excretion by regulating the mechanism of renal reabsorption for uric acid. Gypenosides [81] and ethanol extracts of polygonum sibiricum [82] can lower the expression of URAT1 and GLUT9 protein, affect the mechanism of uric acid reabsorption, and thus regulate uric acid balance. Water extracts of Wudang Cherry can increase the expression of OCT1, OCT2, OCTN1, and OCTN2 protein in HUA animal models, mediate the absorption, reabsorption of various organic cations and carnitine transport, and participate in the excretion of uric acid [83]. *Liriodendron chinense*, commonly known as the Chinese tulip tree, and ethanol extract of the barks of *Liriodendron chinense* (EELC) can significantly increase the excretion of uric acid in hyperuricemic nephropathy (HN) mice, reduce the infiltration of inflammatory factors, and the accumulation of uric acid in the kidney. The progress of HN is reduced by upregulating organic anion transporter 1 (OAT1), OAT3, and ABCG2 protein [84]. Erding granule (EDG) is a kind of Chinese medicine that has the effect of reducing uricemia discovered in recent years. A study has found that 50% ethanol extract (EDG-50) has a significant effect on lowering blood uric acid, which may be related to the downregulation of expression of GLUT9 and URAT1 and upregulation of the expression of OAT1, thus reducing blood uric acid concentration [85]. Berberine can successfully reduce the serum uric acid level of rats with hyperuricemia by increasing the level of uric acid and the excretion fraction of urate in rats [86].

### 5.6. Immune Function Regulation

T cell subsets play an important role in the pathogenesis of gouty arthritis [87]. Isoglycyrrhizin can promote Treg cell induction in vitro and in vivo and inhibit inflammation by reducing IL-2 expression [88]. Simiao powder can improve T cell subsets, upregulate cluster of differentiation (CD3)+ and CD8+ levels, downregulate CD4+ and CD4/CD8 levels, inhibit inflammation, and improve immune resistance [89]. The activation of NLRP3 inflammasome is related to the tilted differentiation of Th subsets for a long time, and it is involved in the occurrence and development of the autoimmune attack. Doliroside A can inhibit both LPS-induced macrophage initiation and inflammatory body activation by inhibiting the caspase-1 dissociation and IL-1*β* secretion [90]. Icariin (ICA) can inhibit nuclear translocation of NF-*κ*B pathway-associated protein and reduces the expression of NALP3 inflammasome in rats [91]. Total glucosides of herbaceous peony (TGPF) can reduce the weight of rats with hyperuricemia nephropathy, reduce serum uric acid (SUA), creatinine (Cr), blood urea nitrogen (BUN), xanthine oxidase (XOD), MCP-1, and TNF-*α*, downregulate kidney URAT1 and GLUT9, upregulate kidney OAT1, and reduce renal pathology associated with hyperuricemia [92]. Compound Shui Niu Jiao granules can significantly inhibit the protein expression of TNF-*α* and IL-8 by injecting sodium urate solution into the articular cavity of model rats with acute gouty arthritis (AGA), reducing inflammatory tissue [93]. Macroporous resin extract of *Dendrobium candidum* leaves is effective in uric acid production inhibition and anti-inflammation in rats with hyperuricemia, and it can inhibit the expression of nuclear factor (NF)-*κ*B, Toll-like receptor (TLR) 4 protein and reduce inflammation [94]. The *Selaginella moellendorffii* prescription (SMP) can significantly reduce the level of uric acid in mice with hyperuricemia and reduce the levels of prostaglandin (PG)E-2, IL-8, nitric oxide (NO), and IL-1 in rats with gouty arthritis. This anti-inflammatory effect may be related to the inhibition of NF-*κ*B p65 nuclear translocation and the expression of NLRP3 protein [95]. An extract of Tu-Teng-Cao (TTC) can inhibit the secretion of cytokines TNF-*α* and IL-6 in synovial fluid of rats, reduce ankle joint damage, and control uric acid and inflammation to treat gouty arthritis [96]. Berberine reduces monosodium urate crystals-induced inflammation by downregulating the expression of NLRP3 and IL-1. The regulation of berberine may be related to the inactivation of NLRP3 inflammasome [97]. Sanmiao wan (SMW) can partially regulate purine metabolism, arginine and proline metabolism, citric acid cycle, phenylpropanoid metabolism, and tryptophan metabolism, reversing the pathological process of hyperuricemia [98]. Modified-Simiaowan (MSW) can protect human umbilical vein endothelial cells (HUVECs) by reducing cell apoptosis and inhibiting the expression of intercellular cell adhesion molecule-1 (ICAM-1) [99]. The ethanolic extract of *Polygonum cuspidatum* can prevent and treat acute gouty arthritis in mice, and its mechanism may be related to the regulation of the expression of the NLRP3/ASC/caspase-1 axis in the gene and protein level [100].

### 5.7. Uric Acid Reduction

Elevated uric acid is the biochemical basis of gout. Uric acid is excreted mainly by filtration, reabsorption, secretion, and other processes involved in transport through the kidneys and intestines. In total, 10% of uric acid is excreted by glomerular filtration and finally discharged from the urine. Totally, 90% of uric acid is reabsorbed by the renal tubules and finally got into blood [101]. Hu et al. found that Simiao pill could promote uric acid excretion and protect the kidney by adjusting urate transporter protein in the kidney of rats with high uric acid [102]. Luteolin and luteolin-4-0-glucoside can act on hyperuricemia mice by lowering mouse urate transporter (mURA)-T1 levels and inhibiting XOD activity [103]. Paeonol is an effective component isolated from *Cortex Moutan*, which can inhibit the expression of proinflammatory cytokines and the activation of NF-*κ*B, significantly decreasing the expression of TNF-*α*, IL-1*β*, and IL-6 in synovium of MSU-induced arthritis (MIA) rats and reducing the formation of uric acid [104]. Compound tufuling oral liquid can reduce gout-induced recurrent joint swelling and pain, significantly reducing serum uric acid (SUA) levels. Besides, the incidence of leukopenia in the treatment group was lower than that in the control group [105]. Polydatin, the natural precursor of resveratrol, can reduce the levels of serum uric acid, creatinine, and urea nitrogen in hyperuricemia rats by interfering with the differential metabolites [106]. Chuanhu antigout mixture (CAGM) and its modified formulation can significantly improve potassium oxonate (PO) induced hyperuricemia in mice, which may be partly due to a decrease in liver XOD and kidney URAT1 levels [107]. Compound Tufuling granules (CTG) have a significant effect on lowering blood uric acid and protecting renal function, which may be related to CTG's ability to regulate the lymph node molecules against inflammation, lower uric acid levels, and protect kidneys [108]. Ethanol extract from *Polyrhachis vicina Roger* (EEPR) can reduce the serum uric acid level of model mice with hyperuricemia. Modified Simiao decoction (MSD) monotherapy is superior to anti-inflammatory drugs and/or uric acid-lowering drugs in treating gouty arthritis, and it can reduce uric acid (UA) and C-reactive protein (CRP) levels; regulate human metabolic disorders; and has no side effects [109–111]. Total flavonoids of *Humulus lupulus* (TFHL) can lower uric acid in hyperuricemia mice by inhibiting the activity of xanthine oxidase (XOD) [112]. Dampness-removing pill (Huashi pills) can inhibit the formation of calculus by regulating urine biochemical indicators and reducing the expression of osteopontin (OPN) in the kidney tissue of rats with kidney stones [113].

### 5.8. Improving Intestinal Flora of Gout Patients

Intestinal flora is associated with the development of many diseases, and intestinal microecology plays an important role in uric acid metabolism and inflammatory response. When the intestinal balance is imbalanced, the status of health will be disrupted, which leads to various diseases, such as gout [114]. After analyzing the diversity of intestinal flora in patients with primary gout and a healthy population, Shi et al. found that *E. faecalis* and xylose-degrading mimics were more abundant in the intestine of patients with gout, whereas *E. faecalis* and Bifidobacterium were absent [114]. Meng et al. found that the application of Chinese herbal medicine to strengthen the spleen and drain turbidity can significantly improve a series of symptoms such as joint redness and pain by reducing the activation of NLRP3 inflammasome in gout patients and regulating the intestinal microecology to increase uric acid excretion [115]. Lin et al. found that the traditional Chinese medicine (TCM) formula, Si-miao-tang, could reduce intestinal apoptosis by inhibiting the expression of NLRP3 inflammatory vesicles, regulating the expression of TNF-*α*, caspase 8, and AIFM1 proteins, and regulating the expression of APOB, LPL, and PPAR*α* proteins to affect lipid metabolism and restore intestinal flora [116]. Gao et al. found that the TCM formula, CoTOL, could reduce body weight and uric acid in mice with hyperuricemia models by regulating intestinal flora [117]. The herbal chicory extract can reduce the activity of key enzymes of uric acid metabolism in hyperuricemic quail, which may be related to regulating intestinal flora and intestinal tight junction protein occludin, increasing the number of beneficial intestinal flora and reducing the number of pathogenic bacteria [118].

### 5.9. Shortcomings of TCM as GA Therapy

#### 5.9.1. TCM Safety for GA Patients

CHM represents an enormous and remarkable treasure trove for new drug development, but the evaluation for the safety of CHM is also required. The oral Chinese medicine formulas have developed quickly and have their own diversity. The safety and efficacy of oral Chinese-patented medicines in treating GA have been confirmed in many clinical studies initiated by Chinese and Western medical researchers [119–124]. Besides, the clinical application of Chinese herbal medicine injection also has attracted attention [125, 126]. Nevertheless, due to the uncertainty of CHM composition, the safety of CHM is still questioned, and the toxic components in CHM have also been described [127]. With the widespread use of TCM worldwide, the safety problems/events of TCM have gradually raised [128]. Especially in recent years, it is reported that serious adverse reactions/events are caused by TCM or its ingredients, such as renal failure caused by Gentian and Liver Pill and liver damage caused by He Shou Wu, and these events have caused great concern both at home and abroad [129–131] and seriously affected the healthy and sustainable development and internationalization of TCM. Some researchers thought that long-term treatment with CHM is still risky, and Chinese medicine still requires massive clinical and basic trials to assess its safety [132, 133].

#### 5.9.2. CHM's Efficacy in Anti-GA Is Still Being Questioned

Great progress has been made in the research of TCM on anti-GA, and some clinical studies have also achieved exciting results [134–138]. Nevertheless, some formulas have a good effect on gouty arthritis, but monotherapy or isolated components can weaken effects or even has no effect at all [139]. The components of CHM are very complicated, but many bioactive ingredients of CHM show only a strong antigouty arthritis effect in vitro, or the antigouty arthritis effect is lost or weakened after purification from the formula. In addition, deficiency of clinical research with high-level evidence seriously restricts CHM's development [140].

### 5.10. Molecular Network Integration for the TCM Modernization TCM in GA Treatment

The pathogenesis of gout is complex. Under the guidance of TCM theory, through long-term application practice, numerous Chinese medicines are effective, safe, cheap, and easily available for the treatment of gout. TCM formulas, consisted of many Chinese traditional herbs, have good efficacy and the least adverse reaction for GA prophylaxis and therapy. Although herbal formulas are widely used in TCM clinical practice, the integration principles based on the theory of TCM are very challenging to identify. In the international community, it is advocated molecular typing of pathogenic genes and the application of precise targeted therapeutic drugs in gout treatment. However, its curative effect is limited, and a single target is not enough to change the prognosis of gout arthritis. Shifting the focal point of anti-GA treatment from accuracy to integration can benefit patients, and it is believed Chinese medicine has the intrinsic strengths for multiingredients strategy [141].

Traditional Chinese medicine has unique advantages in treating gout, but the composition of TCM is complex, and therapeutic targets are various and it is difficult to elucidate the therapeutic targets. Therefore, the specific therapeutic target is an important part of the pharmacodynamic evaluation [142]. Based on modern bioinformatics and network analysis technology, network pharmacology explores the relationship between medicines and gout from the aspects of multitarget and complex diseases, macroscopic and microscopic, fuzzy and visualization, and then clarifies its mechanism of action in treating gout. At the systematic level, network pharmacology promotes drug discovery in an accurate way, establishes a “drug-to-gene-to-target-to-disease subtype” network, and expounds the principle of herbal formula design guided by the theory of TCM, which provides a new way for the modernization of TCM in the future [143, 144].

As an emerging discipline, network pharmacology has made innovative breakthroughs in predicting the genes causing gout and identifying new targets of Chinese medicine. It also provides strong evidence for the development of new drugs, efficacy evaluation, safety evaluation, and quality evaluation of TCM. It will play an important role in all fields of TCM so as to promote the modernization of TCM.

## 6. Conclusions and Prospectives

TCM advocates the preventive treatment of diseases. Under the guidance of TCM theory, targeted rectification can reverse the condition of the disease as soon as possible and prevent the occurrence of diseases. The theory of TCM is often questioned due to its complexity, integrated concept, and symptomatic research. TCM holds that the human body is a complex and dynamic system, which pays more attention to the balance of the internal and external environment. Chinese medicine is a multicomponent, multitarget, and complex mixed system. There are many obstacles in the development of TCM under the background of modern medicine. The unidentified quality of TCM is a shortcoming for it; the necessity of accurate toxicological mechanisms and pharmacodynamic analysis impede the acceptance of TCM in modern times. Besides, antagonistic or synergistic effects of the components in TCM remain unknown. Only after resolving the above problems can TCM truly go abroad. TCM is an essential component of traditional Chinese culture. As Youyou Tu, the first Chinese woman who won the 2015 Nobel Prize in Physiology or Medicine, described, “TCM represents a great treasure house of China. We should make good use of it and create more valuable achievements, so as to bring benefit to human health.”

## Figures and Tables

**Figure 1:** Trends in the treatment of gouty arthritis with TCM. TCM for the prevention and the treatment of gouty arthritis started in Western Han Dynasty and it developed and innovated in Tang Dynasty, Yuan Dynasty, Ming Dynasty, and Qing Dynasty, despite TCM had been doubted constantly. Throughout its history and even it is not valued in modern times, with special reference to the field of gouty arthritis treatment, it still plays a significant role in the treatment of acute and chronic diseases. A great honor and a huge breakthrough for TCM is You-you TU got the 2015 Nobel Prize in Physiology or medicine, and TCM received recognition of the world again. Abbreviations: TCM: traditional Chinese medicine.

**Figure 2:** Chinese medicine herbal formulas include multiple ingredients for wholistic therapy. Herbal formulas consisted of many active ingredients that form the essential units of herbal function, such as the various mechanisms of anti-GA formulas.

**Table 1:** The herbal therapy for GA treatment.

TCM treatment principles	Herbs
Activating blood circulation and eliminating stasis	Chuanxiong Rhizoma (Chuanxiong), Achyranthis Bidentatae Radix (Niuxi), Radix Salviae (Danshen), Persicae Semen (Taoren), Carthami Flos (Honghua), Cortex Moutan (Danpi), Leonuri Herba (Yimucao)

Activating blood circulation and relieving pain	Pollen Typhae (Pohang), *Troopers Dung* (Willingham), myrrh (Moyao), Radix Paeoniae Rubra (Chishao), *Angelicae Sinensis Radix* (Danggui), Panax Notoginseng (Sanqi), *Siphonostegiae Herba* (liujinu)

Clearing away heat and removing dampness	*Phellodendri Chinrnsis Cortex* (Huangbai), *Poria cocos* (Fuling), *Scutellariae Radix* (Huangqin), *Plantaginis Semen* (Cheqianzi), Artemisiae Scopariae Herba (Yinchen), *Atractylodes Lancea* (Cangzhu), *Coicis Semen* (Yiren)

Expelling wind and activating meridians	*Radix Clematidis* (Weilingxian), Radix Angelicae Biseratae (Duhuo), Spatholobus Suberectus Dunn (Jixueteng), Fructuslipuidambaris (Lulutong), *Radix Puerariae* (Gegen), Trachelospermumjasminoides (luoshiteng), *Lumbricus* (Dilong), Ramulus Mori (Sangzhi), *Angelica dahurica* (Baizhi)

**Table 2:** The categories of herbal therapy for GA treatment.

Herbal formuls	Ingredients	TCM efficacy	Provenance	Author
Si-Miao-Wan	Phellodendri Chinensis Cortex (Huangbai), *Atractylodes Lancea* (Cangzhu), *Coix Seed* (Yiren), Achyranthes bidentata (Niuxi)	Clearing away heat and removing dampness	Cheng-fang-bian-du	Zhang bing cheng

Long-Dan-Xie-Gan-Tang	*Gentiana radix* (Longdancao), Glycyrrhiza uralensis (Gancao), *Scutellariae Radix* (Huangqin), *Gardeniae Fructus* (Zhizi), *Rehmannia glutinosa* (Shengdihuang), Radix Bupleuri (Chaihu), Caulis Akebiae (Mutong), *Angelicae Sinensis Radix* (Danggui), *Plantaginis Semen* (Cheqianzi), *Alisma Orientale* (Zexie)	Clearing away heat and dampness; detoxification	Tai-ping-hui-min-he-ji-ju-fang	Liu jing yuan

Bi-Xie-Shen-Shi-Tang	*Dioscoreae Septemlo Bae Rhizoma* (Bixie), *Coix Seed* (Yiren), *Red Poria Cocos* (Chifuling), *Phellodendri Chinrnsis Cortex* (Huangbai), Cortex Moutan (Danpi), *Alisma Orientale* (Zexie), *Talc* (Huashi), *Tetrapanacis Medulla* (Tongcao)	Clearing away heat and removing dampness	Yang-ke-xin-de-ji	Gao bing jun

Qing-re-Hua-Tan-Tang	*Ginseng Radix et Rhizoma* (Renshen), *Rhizoma Atratylodis Mac-rocephalae* (Baizhu), *Poria Poria Cocos* (Fuling), *Glycyrrhizae Radix et Rhizoma* (Gancao), *Red tangerine reel* (Juhong), *Pinellia* (Banxia), *Ophiopogon* (Maidong), *Grass-leaved sweetflag* (Shichangpu), *Fructus Aurantii Immaturus* (Zhishi), *Banksia rose* (Muxiang), *Caulis bambusae* (Zhuru), *Scutellariae Radix* (Huangqin), *Coptis chinensis* (Huanglian), *Arisaema wilsonii Engl* (Nanxing), *Succus bambusae* (Zhuli)	Clearing away heat and removing phlegm	Jing-lue-quan-shu	Zhang jing yue

Dang-gui-Nian-tong-Tang	Notopterygii Rhizoma Et Radix (Qianghuo), *Ginseng Radix et Rhizoma* (Renshen), Sophorae Flavescentis Radix (Kushen), Cimicifugae Rhizoma (Shengma)*, Radix Puerariae* (Gegen)*, Atractylodes Lancea* (Cangzhu), Glycyrrhiza uralensis (Gancao)*, Scutellariae Radix* (Huangqin), Artemisiae Scopariae Herba (Yinchen)*, Saposhnikoviae Radix* (Fangfeng)*, Angelicae Sinensis Radix* (Danggui)*, Anemarrhenae Rhizoma* (Zhimu), *Alisma Orientale* (Zexie)*, Polyporus umbellatus* (Zhuling)*, Atractylodes Macrocephala Koidz* (Baizhu)	Dispelling heat and dampness, dispelling wind and relieving pain	Dan-xi-xin-fa	Zhu dan xi

Yin-Chen-Wu-ling-San	Artemisiae Scopariae Herba (Yinchen), *Alisma Orientale* (Zexie), *Polyporus umbellatus* (Zhuling), *Atractylodes Macrocephala Koidz* (Baizhu), *Poria Cocos* (Fuling), Cinnamomi Ramulus (Guizhi)	Clearing away heat and removing dampness	Jin-gui-yao-lue	Zhang zhong jing

Ba-Zheng-San	Radix Rhei Et Rhizome (Dahuang), *Plantaginis Semen* (Cheqianzi), Dianthi Herba (Qumai), Polygoni Avicularis Herba (Bianxu), *Gardeniae Fructus* (Zhizi), Caulis Akebiae (Mutong), Glycyrrhiza uralensis (Gancao), *Talc* (Huashi)	Clearing away heat and purging fire, promoting urination	Wai-ke-zheng-zong	Chen shi gong

Wu-Wei Xiao-Du-Tang	*Lonicerae Japonicae Flos* (Jinyinhua), Chrysanthemi Flos (Juhua), *Dandelion* (Pugongying), *Violsse Herba* (Zihuadiding), *Begonia fimbristipula* (Zibeitiankui)	Clearing away heat and toxin, resolving carbuncle and node	Wai-ke-zheng-zong	Chen shi gong

Xuan-Bi-Tang	*Stephaniae Tetrandrae Radix* (Fangji), Amygdalus Communis Vas (Xingren), *Talc* (Huashi), *Forsythiae Fructus* (Lianqiao), *Gardeniae Fructus* (Zhizi), *Coicis Semen* (Yiren), Arum Ternatum Thunb (Banxia), *Silkworm excrement* (Cansha), Phaseoli Semen (Chixiaodou)	Clearing away heat and dampness, promoting channels and collaterals	Wen-bing-tiao-bian	Wu ju tong

Dang-Gui Shao-Yao-Tang	*Angelicae Sinensis Radix* (Danggui), *Paeoniae Radix Alba* (Baishao), *Poria Cocos(Schw),, Wolf* (Fuling), *Atractylodes Macrocephala Koidz* (Baizhu), *Alisma Orientale* (Zexixe), Chuanxiong Rhizoma (Chuanxiong)	Invigorating the spleen, nourishing the blood and regulating the liver	Jin-gui-yao-lue	Zhang zhong jing

## Data Availability

The data used to support the findings of this study are available from the corresponding author upon request.

## Abbreviations

GA: Gouty arthritis
TCM: Traditional Chinese medicine
CHM: Chinese medicine
MSU: Monosodium urate
CAMs: Complementary and alternative medicines
WHO: World Health Organization
IL-6: Interleukin-6
VAS: Visual Analogue Scale
TNF-*α*: Tumornecrosis factor-*α*
AGA: acute gouty arthritis
Bcl-2: B-cell lymphoma
GSH-Px: Glutathione peroxidase
SOD: superoxide dismutase
B C: Before Christ
MDA: Malondialdehyde
Nrf2/HO-1: Nrf2-mediated induction of heme oxygenase-1 (HO-1)
SIRT1: Sirtuin1
miR-34a: MicroRNA 34a
ROS: Reactive Oxygen Species
LPS: Lipopolysaccharide
NLRP3: NOD-like receptor (NLR) family, pyrin domain-containing protein 3
ERK1/2: Extracellular signal regulate kinase 1/2
Nrf2: Nuclear factor erythroid-2 related factor 2
COX: Cyclooxygenase
MPO: Myeloperoxidase
XOD: Xanthine oxidase
ADA: Adenosine deaminase
IFN: Interferon
MIP-1a: Macrophage inflammatory protein-1a
PKA: Protein kinase A
OAT3: Organic anion transporter 3
HUA: Hyperuricemia
TLR 4: Toll like receptor 4
NO: Nitric oxide
(PG)E-2: Prostaglandin E-2
MIA: MSU-induced arthritis
SUA: Serum uric acid
UA: Uric acid
RBXG: Rebixiao granules
MSU: Monosodiumurate
GSH-Px: Glutathione peroxidase
GSH: Reduced glutathione.
UAN: Uric acid nephropathy.
